RETRACTED

# Knowledge, attitude and practices in relation to prevention and control of schistosomiasis infection in Mwea Kirinyaga county, Kenya

**DOI:** 10.1186/s12889-016-3494-y

**Published:** 2016-08-18

**Authors:** J Mwai, S Njenga, M Barasa

**Affiliations:** Kenya Medical Research Institute, Box 54840-00200, Nairobi, Kenya

**Keywords:** Knowledge, Attitude, Practice, Prevention, Control, Schistosomiasis, Mwea

## Abstract

**Background:**

Schistosomiasis remains a major public health problem in Kenya. Inadequate knowledge, attitudes and practices (KAP) on causative factors are some of the critical factors for the increased prevalence. The study assessed KAP on the control and prevention of schistosomiasis infection in Mwea division, Kirinyaga County-Kenya. Four hundred and sixty five house-hold heads were enrolled in this study by use of simple random sampling technique.

**Methods:**

The study employed an analytical descriptive cross sectional design utilizing both quantitative and qualitative data collection methods. A pretested structured questionnaire, Focus Group Discusions (FGDs) and Key Informant Interviews (KII) guides were used for data collection. Descriptive statistics and Chi square tests and Fisher’s exact tests were computed where applicable. Data from the FGDs and KIIs were analyzed using NUID.IST NUIRO.6 software.

**Results:**

Significant associations between knowledge and demographic factors i.e. age (*p* = 0.011), education level (*p* = 0.046), were reported. Handwashing after visiting the toilet (*p* = 0.001), having a toilet facility at home (*p* = 0.014); raring animals at home (*p* = 0.031), households being affected by floods (*p* = 0.005) and frequency of visits to the paddies (*p* = 0.037) had a significant association with respondents practices and schistosomiasis infection. Further significance was reported on households being affected by floods during the rainy season (*p* < 0.001), sources of water in a household (*p* < 0.047) and having a temporary water body in the area (*p* = 0.024) with increase in schistosomiasis infection. Results revealed that respondents practices were not significantly associated with gender (*p* = 0.060), marital status (*p* = 0.71), wearing of protective gear (*p* = 0.142) and working on the paddies (*p* = 0.144).

**Conclusions:**

This study reveals that knowledge about the cause, transmission, symptoms and prevention of schistosomiasis among the Mwea population was inadequate, and that this could be a challenging obstacle to the elimination of schistosomiasis in these communities. Due to various dominant risk factors, different control strategies should be designed. Therefore, there is a need for integrated control programme to have a lasting impact on transmission of schistosomiasis infection. Control programs like mass drug administration need to go beyond anti-helminthic treatment and that there is a need of a more comprehensive approach including access to clean water, sanitation and hygiene. School and community-based health education is also imperative among these communities to significantly reduce the transmission and morbidity from schistosomiasis.

RETRACTED

## Background

In 2001 a resolution was passed during the 54th World Health Assembly (WHA) with the target (for member states) to regularly administer anthelmintic drugs to at least 75 % and up to 100 % of all school-aged children at risk of morbidity due to schistosomiasis by 2010 [1]. In the same year, the World Health Organization (WHO) assembled an expert committee to refine the global strategy for the prevention and control of schistosomiasis. Since then, millions of school-aged children have received praziquantel against schistosomiasis [2]. Even though it has limitations because older population segments are insufficiently addressed, and hence new knowledge on prevention and control of schistosomiasis infections is minimal [2].

In Kenya, more than 6 million people, or approximately 23 % of the total population, are infected with urinary or intestinal schistosomiasis [1]. In 2005, Kenyan Ministries of Health and Education initiated a parasite control programme with the aid of Japan International Co-operation Agency (JICA) and Kenya Medical Research Institute (KEMRI). The programme was targeting S. mansoni and Soil transmitted helminthes (STHs) in school age children. After sensitizing and educating the community health officers and education officers in the district, 43,928 school age children from 86 schools were de-wormed with praziquantel and albendazole by trained school teachers [3]. Prior to the de-worming, baseline prevalence and intensity of parasitic infections were determined through examination of stool samples of class three children (age range 9–14 years). A follow up study of five cohort primary schools was carried out to monitor the effectiveness of the control programme for four consecutive years. The prevalence of the parasitic infections in the five cohort schools was 38 % for S. mansoni before treatment [4]. However, there was an overall parasitic re-infection rate of 16 % for S. mansoni, 6 months after treatment. The trend of re-infection continued after treatment to 22 % in the second year, 31 % in the third year and 17 % in the fourth year [4]. Although the program achieved significant results, there is a continuous challenge of disease re-establishment after completion of program [5]. Mwea irrigation scheme in Kirinyaga County, where transmissions of schistosomiasis, is relatively high has a prevalence of 47.4 % [3].

RETRACTED

Knowledge, Attitudes and Practices in relation to the disease are critical in establishing effective control measures. However, data on the knowledge, attitude, and practices (KAP) of populations in endemic areas in Kenya with regard to schistosomiasis are not available. Community awareness and involvement are considered as one of the cardinal tools for the success and sustainability of any disease control programme [3]. Within this context, the present study aims to evaluate the KAP towards schistosomiasis in the Mwea Population. It is hoped that the findings will provide new information about the schistosomiasis-related KAP of the targeted population, and will add new insights about the prevention and control of this devastating disease in Kenya.

## Methods

### Study area

The study was conducted in Mwea irrigation scheme located in Kirinyaga County, central Kenya. Administratively, the new upgraded Kirinyaga County has two districts (Mwea East and Mwea West). The county is located about 100 km north east of Nairobi, Kenya. It covers an area of 513 km2 and it is estimated to have 51,444 households and a total population of 176,261 persons. The mean annual rainfall in this area is in the range of 1200–1600 mm per year and varies by the time of year. Mwea West district, where the study was conducted has two locations (Kangai and Thiba) and seven villages. The main socio-economic activity in this area is rice farming, which is done by gravity flow irrigation using water from river Thiba and Nyamindi. Mwea west district is endemic for both S. mansoni and Soil transmitted helminths (STH).

### Study design

The study employed descriptive cross-sectional design adopting both qualitative and quantitative data approaches for assessing Knowledge, Attitude and Practices on schistosomiasis prevention and control in Mwea division of Kirinyaga Sub County.

### Study population

The division was selected based on schistosomiasis endemicity in the area after doing a consultation with the District Public Health Officer and previous studies conducted in the area in the control program [3]. The study population will be selected on the basis of availability during the time of study.

### Sample size determination

The minimum sample size will be computed using the formula by Fischer et al. [6].

The current prevalence is unavailable, thus an assumed prevalence of 50 % will be used in the computation of the minimum sample size required for this study.

$$ \mathrm{n}=\frac{{\mathrm{z}}^2\upalpha \mathrm{p}\mathrm{q}}{{\mathrm{d}}^2} $$ Where

Z_α_: = standard normal deviate = 1.96
p: = estimated prevalence. = 0.5 (50 %)
q: = (1 − p) = 0.5
d: = (Precision) = 0.05

$$ \mathrm{n}=\frac{(1.96)^2(0.50)(0.50)}{0.05^2} $$ n = 384.16 approximately 385 participants

385 × 1.2 (design effect) = 461 participants is the minimum sample size required for the study.

RETRACTED

### Sampling procedure

Three villages were purposively sampled based on high schistosomiasis prevalence for the study [3]. The number of households to participate, in each of the three villages were selected with a probability proportionate to their sizes and Mianya which has 1200 households was represented by 301 households, Murubara has 500 and was represented by 126 and Mbui Njeru which has a total of 135 households was represented by 34 households.

### Selection of households

In the quantitative component, simple random sampling technique was applied to select the households from each village. The number of households per sub-location depended on the household sizes. The household heads were interviewed in each household, in the absence of the household head an adult representative was interviewed using the structured questionnaire.

### Questionnaire

An interviewer based questionnaire was used for the household heads. Issues pertaining to socio-demographic characteristics, water usage and sanitation, knowledge, attitudes and practices related to schistosomiasis infection, housing factors (such as type of construction of the house, type of floor inside house, sanitary conditions, waste disposal, acceptability and willingness to use the current preventive and control measure was used. Questionnaires were administered with both closed ended and open ended questions to capture elements of quantitative and qualitative data respectively. The questionnaire was administered using the local language and translated to English and Kiswahili.

### Qualitative data

#### Key informant interviews

Stratified purposive sampling technique was used to select key personalities i.e. local administration, head teachers, opinion leaders, religious and group leaders and health officers. In each village, schools were selected for each division and the headmasters for the selected schools were interviewed in any one school. Purposive selection was done in the village. The village elders, an area member of parliament or councilors, health officers in the local health facilities and church or mosque leaders were also interviewed. At least 10 key informant interviews were conducted in the three administrative locations, totaling up to 30 interviews. The key informant guide that was developed was pre-tested and amended accordingly and used to interview the above selected participants in various aspects. The guide was used to explore the individual knowledge, attitude and practices on schitosomiasis infection. The KII guide helped in exploring the insights of the real issues in regard to factors influencing the prevention and control of schistosomiasis infection from the informants.

RETRACTED

A total of 18 in-depth interviews were conducted with opinion leaders from three administrative locations. Fourteen of the participants were male and four female.

The respondents mean age was 50, the youngest was 26 years old and the oldest was 75 years old. Majority (6) of respondents were farmers and teachers were three while three were village elders and three social group leaders with three business people. All (18) respondents were Christians, 17 were married and one was single.

### Focus group discussions

Focus group discussions were conducted and led by trained moderators and note-takers fluent in the local languages on the above selected participants. The researcher developed themes and sub-themes on the subject of discussion. The themes and sub-themes developed were used to probe the members, while the note takers were recording gestures, assent, expressions, and other non-verbal information that maybe coming out. An evaluation was done at the end of the meeting by the researcher to validate the information collected. Discussions were gathered on two digital voice recorders and transcription were done by voice recognition software called Dragon voice recognition then typed into Ms Word and analyzed using the NUDI.ST NUIRO.6 software.

A total of 12 FGDs were done in all the three administrative locations, with each of the administrative locations having four FGDs each. The participants were asked to attend a specially arranged session of 30 to 45 min for a focus group discussion. The FGDs participants included single sex adult (36 years and above) and youth (18 to 35 years) male and female participants of homogenous characteristics. The FGDs were further categorized into gender (male youth and female youth and female adult and male adult). The adults had to be between 36 years of age and above. There was no exclusion in terms of language for this category Study participants were randomly selected from pools of individuals that met the inclusion criteria. The youth, whether male or female had to be between 18 and 35 years of age and able to speak either English or Swahili. Each FGD contained a minimum of 8 and a maximum of 12 participants. Community health workers, familiar with the villages, helped to mobilize participants for the study. Further screening was done on site to make sure that participants met the inclusion criteria before obtaining consent, and that they were fully representative of the different villages.

RETRACTED

### Quality assurance

Quality assurance measures included training enumerators and data entry clerks on the survey instruments, field testing with a special focus on a ‘real-life’ situation, as much as possible so as to improve the process and to enhance the understanding of the study team. Field supervisors were also engaged to immediately review questionnaires on a daily basis and to rectify any inconsistencies that may arise. Data Cleaning was a multi-stage process. The data was cleaned immediately after data entry in MS Access, data was continually exported to excel and fed into SPSS during analysis until the final report was completed.

### Data management and analysis

Quantitative data collected was entered into the Ms Excel and Access software. Statistical analysis was done after data validation. Descriptive statistics including mean, or median, frequencies and proportions were appropriately generated. Chi square test was used to test associations between variables. Bivariate analysis was performed to identify the factors significantly associated with the KAP variables among the studied population. A *P* value of <0.05 was considered to be statistically significant.

Data collected from qualitative interviews was transcribed verbatim into Microsoft Word. The research team then checked the consistency of the transcripts against the audio files to ensure accuracy of the transcribed files. The cleaned transcripts were then imported into qualitative text analysis software NUID.IST NUIRO.6 This software allowed the data to be coded systematically. Qualitative data was analysed using content and thematic analysis to identify emerging themes. The process of analysis involved familiarization with the data, development of initial codes based on the research questions and issues emerging from data, refinement of codes and their allocation to broad themes. Data was then stored in electronic storage devices like DVDs, USB, files containing the data were encrypted and access was only authorized PI to ensure quality control.

## Results

### Socio-demographic characteristics of the respondents

The results indicating socio-demographic characteristics of the respondents are presented in Table 1. Out of the 400 and 65 respondents, there was a higher number of females (63.9 %) while males were 36.1 % in the three divisions, with a significant difference between the genders. There were also significant differences in the categories of age, marital status, religion, occupation and education level. The majority (70.0 %) of the participants were married compared with 30.0 % who had never married. In the selected communities, the majority of the residents were farmers 79.1 % while less that 1.0 % were unemployed. Primary-educated residents accounted for 67.0 %, while the rest had either, no formal education, secondary education or postsecondary. Notably, the majority of residents (99.6 %) were predominantly Christians with Muslims and others constituting only 0.2 %.

RETRACTED

**Table 1:** Socio-demographic characteristic of respondents

Variable	Response	No. of respondents (*N* = 465) Percentage (%)
Gender	Male	168 (36.1 %)
	Female	297 (63.9 %)
Marital status	Married	371 (70.0 %)
	Single	45 (13.8 %)
	Divorced	23 (7.9 %)
	Widow	20 (6.3 %)
	Widower	6 (2.0 %)
Religion	Christian	463 (99.6 %)
	Muslim	1 (0.2 %)
	Other	1 (0.2 %)
Level of education	No Formal Education	34 (7.3 %)
	Primary Education	311 (66.9 %)
	Secondary Education	107 (23.0 %)
	Post Secondary	11 (2.4 %)
Occupation	Public Servant	4 (0.9 %)
	Farmer	368 (79.1 %)
	Business	32 (6.9 %)
	Informal Employment	59 (12.7 %)
	Not Employed	2 (0.4 %)
Age group (years)	17–30 years	166 (35.8 %)
	31–40 years	126 (27.1 %)
	41–50 years	60 (12.8 %)
	51–60 years	49 (10.6 %)
	61–70 years	40 (8.4 %)
	71–80 years	18 (3.8 %)
	81–90 years	6 (1.3 %)

### Knowledge about schistosomiasis, symptoms, transmission, prevention and control among Mwea population

From the analysis, over half of the participants (58.71 %) indicated that the most common disease in the area was schistosomiasis. Majority of the respondents (92.9 %) stated that they were aware of schistosomiasis. A third of the participants (39.87 %) indicated health workers as the main source of information. Another third of the participants (30.51 %) mentioned stomach ache as the most common sign and symptom of schistosomiasis. Approximately 41 % of the respondents stated that the disease was transmitted through contact with infected water while about 14.04 % did not know the medium of transmission. Study results reveal that majority of the respondents or a member of their household (70.97 %) had suffered from schistosomiasis. Slightly above a third of the participants (34.49 %) indicated the use of toilet facility as a way of preventing schistosomiasis, and for those already infected over half of the respondents (51.79 %) indicated that prescribing to schistosomiasis medication would avoid the risk of re infection. With regard to intervention strategies for schistosomiasis, slightly below half of the respondents (49.25 %) indicated that community intervention programmes existed, with a third of the participants (31.6 %) stating that the intervention programmes were government initiatives as indicated on Table 2.

RETRACTED

**Table 2:** Knowledge about schistosomiasis, symptoms, transmission, prevention and control among Mwea population

Questions	Response	n (%)
Have you heard of schistosomiasis	Yes	432 (92.90)
	No	32 (6.88)
	No Answer	1 (0.22)
Have you or any member of your household suffered from schistosomiasis?	Yes	330 (70.97)
	No	135 (29.03)
In your Knowledge, have there been any community intervention programmes on schistosomiasis prevention and control in this area?	Yes	229 (49.25)
	No	236 (50.75)
If yes, which programmmes are these?	Government Programmes	147 (31.6)
	NGO Programmes	59 (12.7)
	FBO Programmes	0 (0)
	Community Initiated	19 (4.1)
	Individual Initiated	2 (0.4)
	Don’t Know	8 (1.7)
	NA	230 (49.5)
What is the Common Disease in this area?		
	Frequency	Percent
Bilharzia	273	58.71
Malaria	163	35.05
Diarrhoea	8	1.72
Don’t know	5	1.08
N/A	2	0.43
Other	14	3.01
Total	465	100.0
How can a person prevent him/herself from getting Schistosomiasis?		
Not working in rice fields	77	15.71
Not using other person’s belongings	13	2.65
Stepping or walking on dirty water	94	19.18
Washing hands	80	16.33
Using the toilet facility	169	34.49
Wearing of shoes	57	11.63
Total	490	100
Which of the following signs and symptoms did you or members of your family experience?		
Stomach ache	285	29.5
Vomiting	115	11.9
Diarrhea	221	22.88
Bloody Stool	212	21.95
Swollen Stomach	27	2.8
Abdominal Pain	106	10.97
Total	966	100
How can a person who is already infected with Schistosomiasis reduce their risk of re infection?		
Prayer	4	1.02
Practice good sanitation	169	43.11
Putting on of gumboots while in the pad	16	4.08
Those already infected to take medicine	203	51.79
Total	392	100
When are you likely to get Schistosomiasis?		
Wading, bathing or swimming in infected	212	35.1
Working/rice planting in rice paddies	309	51.16
Interaction with infected persons	18	2.98
Not using the toilet facility	64	10.6
Use of other persons’ personal belonging	1	0.17
Total	604	100
Source of Information on Disease		
Media	37	5.9 %
Health Workers	250	39.87 %
Family	118	18.82 %
Friends, Peers	111	17.7 %
Religious Leader	9	1.44 %
Teacher	61	9.73 %
Community Baraza	32	5.1 %
Campaigns	9	1.44 %
Total	627	100 %

### Association of awareness of the participants on schistosomiasis with some demographic factors

The study results on the association between demographic characteristics and awareness on schistosomiasis are as presented in Table 3. The results revealed that awareness on schistosomiasis was significantly associated with age (*p* = 0.011) and education level (*p* = 0.046). However the results revealed that awareness on schistosomiasis was not significantly associated with gender (*p* = 0.060) and marital status (*p* = 0.71).

RETRACTED

**Table 3:** Association of awareness of schistosomiasis with some demographic factors

Factors	Awareness		Total	Statistical Significance
	Yes n (%)	No n (%)		
Gender				
Male	158 (94.0)	7 (6.0)	168 (100)	*p* = 0.060
Female	268 (90.2)	29 (9.8)	297 (100)	
Age				
17–30	144 (86.7)	22 (13.3)	166 (100)	*p* = 0.011
31–40	123 (97.6)	3 (2.4)	126 (100)	
41–50	53 (88.3)	7 (11.7)	60 (100)	
51–60	46 (94)	3 (6)	49 (100)	
61–70	37 (93.9)	2 (6.1)	40 (100)	
71–80	18 (100.0)	0 (0.0)	18 (100)	
81–90	4 (66.7)	2 (33.3)	6 (100)	
Education				
Not Educated	30 (88.2)	4 (11.8)	34 (100)	*p* = 0.046
Primary	304 (97.7)	7 (2.3)	311 (100)	
Secondary	107 (100.0)	0 (0.0)	107 (100)	
Post Secondary	8 (72.7)	3 (27.3)	11 (100)	
Marital Status				
Married	344 (92.7)	27 (7.3)	371 (100)	*p* = 0.071
Single	39 (86.7)	5 (13.3)	45 (100)	
Divorced	19 (82.6)	4 (17.4)	23 (100)	
Widow	20 (100.0)	0 (0.0)	20 (100)	
Widower	5 (83.3)	1 (16.7)	6 (100)	

### Qualitative data presentation

#### Assessment of knowledge and awareness

##### Avenues of information

The FGDs with community members revealed that the majority of the participants had heard about schistosomiasis before. The sources of information included schools, posters, radio and community gatherings (*baraza*), with the health workers the most mentioned. A 37-year-old male casual labourer (informal employment) from Mianya said, *“I heard about it through the community health workers, they normally visit us a lot especially when there are barazas at the chief’s camp for health talks especially on schistosomiasis.”*

### Preferred sources of information

With regard to spreading information about schistosomiasis, participants mentioned a few sensitization methods that they felt would work best in their community: a 40-year-old female farmer from Murubara said: *“Door to door is best because the village elders know each and every one of their village and they can do it easily*…*.”* A 37-year-old male farmer in Mianya said: *“I wish they can use billboards up to those rural areas it is the best one because you see as you walk.”*

### Knowledge about schistosomiasis

Adult male FGDs indicated that some of the common diseases in the area were (as mentioned by participants); *Schistosomiasis, Malaria, and high blood pressure and the* main symptoms (as mentioned by participants); Urinating blood, blood in stool, stomach ache, head ache, dizziness and joint aches. Our study revealed that the majority of the participants felt they did not have adequate information about schistosomiasis. A 30-year-old female business owner from Mbuinjeru said: *“Some are informed while others are not, depending on the literacy level. If you didn’t go to school then you can’t be informed about it.”* A 26-year-old male youth in Mianya said: *“Me personally, I don’t think that am well informed about it, because I only know that it is being caused by snails in the infested areas but what about the symptoms and the medications? I don’t know.”*

RETRACTED

Some of the participants had some information on how the disease can be prevented. For example, a 27-year-old adult female from Mbuinjeru said: *“I think by washing hands before eating, entering the rice paddies with gum boots can help in prevention.”* A male youth from Murubara: *“For example, if I apply jelly oil before entering the rice paddies then I won’t be infected.”*

But lack of knowledge also turned out to be expensive for the community economically. This was echoed by one of the male respondents from the key interviews who reported that ‘*due to lack of knowledge the community do face problems when they are infected with Schistosomiasis for it often causes death and also a lot of energy is lost in terms of finances, much time is consumed hindering one from participating in economic growth and it impairs growth in children’* 43 years old village elder from Mbuinjeru division.

### At risk groups

It was the general view of participants that there is no particular gender or age that is more at risk compared with others. They attributed this to modernization where both women and men do more or less the same tasks and have the same levels of exposure as explained by a 55-year-old female farmer in Murubara *“I think both male and female. Because nowadays, people believe that it is gender equality. What men can do, ladies also try.”* This was echoed by a 37-year-old farmer from Mbuinjeru, *“As for me, I think anybody can get infected by this disease (schistosomiasis), whether it’s a child or an adult and especially those people whose main work constantly involves water.”* A few however, bearing in mind gender roles, felt that a particular gender was more at risk *“For me, if I may reflect back on how we grew up, men*…*, male children were the people who were really affected by schistosomiasis; I didn’t know any girl suffering from schistosomiasis; I can’t tell whether they were infected since I did not observe it—perhaps they hid it as girls. So it is us men who would realize that we were passing out blood or victims of bilharzia. The reason why we are mostly affected is that we expose ourselves in areas having water when we go to graze animals or when we are playing while girls are always at home.”* said a 44-year-old farmer from Mbuinjeru. FGD youth female indicated rice farmers, and children as the group that tends to get the disease more with challenges faced from the disease (as mentioned by participants); Weakness, unable to eat, going to the toilet many times, some people become bed ridden. Though adult male FGDs showed that everybody was at risk of getting the disease.

RETRACTED

### Assessment of attitudes

One of the factors that the participants mentioned and that could pose as a barrier in schistosomiasis control is the attitude of community members toward those infected with the disease. A 42-year-old male farmer in Murubara said: *“They can judge you and mistake it for other diseases like HIV.”* A 47-year-old female in Mbuinjeru put it succinctly: *“when you suffer from those symptoms like diarrhea and swollen stomach, they think that you are HIV positive.”* A female youth in Mianya said: *“I think when you become sick, there are things you can’t share with your spouse like blankets.”*

The youth female FGDs thought that toilets should be build, they should come together and build toilets in the paddies as a community and that the government needs to be more involved by building more latrines, taking care of existing latrines and educating the community on health education more often. A 42 years old farmer in Mianya said *“our people don’t like using latrines in the paddies, majority would rush home to use latrines and some do not mind they just diarrhea in the paddies.”*

### Seeking treatment

The majority of the participants thought that treating schistosomiasis is very expensive. The youth female discussions indicated that seeking treatment is costly and its time consuming. Participants indicated visiting the health facility for treatment and drugs but some opted to use herbal treatment which they found cheap. Community members opted to optimize the door to door campaign by the health worker as reported by a 40-year-old administrator from Mianya, ‘*the community have advanced a step forward in the recent days out of the tireless activities of our community health workers who go door to door to campaign and teach our community on general health issues and even give our children dewormers’*.

### Susceptibility and severity

More than half of the participants were of the opinion that schistosomiasis is a serious disease, and that their activities exposed them to infection. These sentiments were reflected by a 25-year-old female youth in Mianya division *“Where I come from it is a problem because, next to our home we have a river. People swim there* …*.”* A 35-year-old female from Mbuinjeru went on to elaborate *“Shistosomiasis is not a joke, reason being that it also brings with it headache, diarrhea of bloody stool, and as you urinate blood you end up losing a lot of blood. So it comes along with many infections to your body. You are always weak even standing up to walk becomes a problem.”* Similar thoughts were echoed by a 40-year-old male administrator from Murubara. *“It’s very serious because any disease can kill if not treated in time, so according to me schistosomiasis can kill and therefore it’s a very serious disease.”*

RETRACTED

### Assessment of practice

#### Use of sanitation facilities and hand washing (*p* = 0.014, *p* = 0.001)

Most of the community members thought that they are the main cause of spreading the disease. For example, one of the respondent who is a farmer aged 60 years from Murubara Division reported that ‘*the community in large numbers do not use pit latrine and they usually dig shallow holes which after filling they take a long time to prepare another one’.* A village elder who is 43 years old from Mianya also lamented that *‘the community around me do use toilet but in most cases they forget to wash their hands after visiting the toilet which is a link to one of the diseases like diarrhea’.*

This was further echoed by one of the respondent from the key informant interviews who reported that*’ there is need for the community to be sensitized on how to use the toilet facilities for not many do wash hands after visiting the toilet.’72* year old retired teacher from Murubara.

Seventy five year old chairman in one of the organizations reported that’ *most of the community members working in paddies have no toilets, hence they go to the canals or in the rice fields to relieve themselves’.* A local administrator to the area also lamented that *‘I would say that the community within my area of jurisdiction are conversant with using toilet for about 60 % residential do each have a toilet facility only that some sense of hygiene need be conveyed to many because about 40 % of these people do not remember to wash their hands after visiting the toilet before eating.*

### Wearing protective gear (*p* = 0.142)

On wearing of protective gear, a 51-years-old administrator from Mbuinjeru division reported that ‘*in actual fact, practices of wearing protective gears while in the rice paddies is inevitable unless maybe they may be introduced to farmers in future for there has never been such commodities ever since rice farming was invented in Mwea scheme’.*

A 56-year-old Director at a local factory reported that’ t*hey are not needed most people do not know the importance of using protective wears they say they are too heavy e.g. gum boots and hand gloves will make them work slowly in paddies and they are so expensive’.*

One of the respondents aged 26 also reported this on wearing protective gear *‘the community at large do not wear any protective gear because the paddies are very deep’.*

RETRACTED

### Household compound affected by floods (*p* = 0.005) and water for use in the household

A common practice by the community members included, fetching water for household use from canals, drainage, paddies this was from the youth male FGDs. On households being affected by floods, one of the key informants reported that *‘most of the area is flooded with water in rainy season. Many people do not use toilet facilities’* a 50 year old female farmer from Mianya division. Another respondent who is 40 years of age from also added that ‘*many toilets within the region are 3 ft or 4 ft they stay for 3 months in dry spells but during rainy season they are over flown with water all over the village’.*

A 33 years old male instructor from Murubara reported that ‘*the area is swampy and you dig 3 ft deep and after the rainy season water floods all over the community making it dirty. Therefore the water available becomes contaminated hence wasted for there is no piped water.*

### Association between practices and having suffered from schistosomiasis infection

Table 4 indicates the relationship between practices and having suffered from schistosomiasis infection. There was an association (*p* = 0.037) between frequency of visits to the paddies and having suffered from schistosomiasis infection. There was a significant association between washing of hands after visiting the toilet and having suffered from schistosomiasis infection (*p* = 0.001). Further, the results show that having suffered from schistosomiasis infection had a significant association with having a toilet facility at home, (*p* = 0.014); raring animals at home (*p* = 0.031) and household being affected by floods (*p* = 0.005). Study indicate no significant association between working in the paddies (*p* = 0.144), not wearing protective footwear (*p* = 0.142) and having suffered from schistosomiasis infection.

**Table 4:** Distribution of respondents’ practice and having suffered from schistosomiasis infection

Factors	Having suffered from Schistosomiasis infection		Total n (%)	Statistical Significance
	Yes n (%)	No n (%)		
Working in the paddies				
Yes	325 (74)	113 (26)	438 (100)	*p* = 0.144
No	17 (65)	10 (35)	27 (100)	
Frequency of visiting paddies				
Frequently	284 (76)	91 (24)	375 (100)	*p* = 0.037
Rarely	38 (61)	25 (39)	63 (100)	
Wearing protective footwear while in the paddies				
Yes	5 (56)	4 (44)	9 (100)	*p* = 0.142
No	320 (74)	111 (26)	431 (100)	
Handwashing after toilet visiting				
Yes	176 (64)	99 (36)	275 (100)	*p* = 0.001
No	160 (84)	30 (16)	190 (100)	
Sanitation facility available at home				
Yes	323 (73)	119 (27)	442 (100)	*p* = 0.014
No	20 (87)	3 (13)	23 (100)	
Raring Animal at home				
Yes	178 (80)	46 (20)	224 (100)	*p* = 0.031
No	168 (70)	73 (30)	241 (100)	
H/Hold compound affected by floods				
Yes	258 (78)	75 (22)	333 (100)	*p* = 0.005
No	84 (64)	48 (36)	132 (100)	

RETRACTED

## Discussion

Study findings showed that 39.87 % of the respondents indicated that they had heard about the disease from the healthcare personnel. However, a study in Senegal [7] showed low awareness of intestinal schistosomiasis among the population. Despite 7 years of health education interventions using a diversity of communication outlets including radio, television and posters, a previous study in Senegal revealed that although 86 % of the respondents stated that they had heard about schistosomiasis, only 30 % had adequate knowledge about the symptoms and modes of transmission of the disease [7]. The present study revealed poor knowledge about the modes of transmission and preventive measures of schistosomiasis; with 34.49 % of the respondents indicating that use of toilet facility would prevent one from getting schistosomiasis infection. In western Kenya, a previous study found that some of the participants knew snails and poor sanitation contributed to the spread of the disease, but lacked understanding of the transmission cycle [7]. Hence, it is clear that the lack of this knowledge among the targeted population may create an additional burden and cost for controlling the disease and may cause the failure of the schistosomiasis eradication programme.

Although the majority of the respondents had heard about schistosomiasis, the results showed that awareness about the symptoms, ways of transmission and preventive and control measures among the participants was generally poor. The present study was carried out in endemic areas that underwent the active control and prevention surveillance by Japan International Cooperation Agency (JICA together with GoK line ministries (MoH, MoE) which may explain why 92.90 % of the respondents had heard about the disease. This is also consistent with the finding that 70.97 % of the respondents had declared history or a member of their household having suffered from shistosomiasis which supports the endemicity of infection in these communities. Study findings revealed that 28.50 % of the respondents mentioned stomachache as the main signs and symptoms. Conversely, previous studies from Brazil and Ethiopia reported diverging information where the majority of the subjects were able to associate these symptoms with the infection [8, 9]. Similarly, it is also worth noting that knowledge about the symptoms of schistosomiasis among the respondents was negligible, as only 22.88 % of them mentioned diarrhea and 21.95 % blood in stools. This could be attributed to the disease being frequently confused with other intestinal infections exhibiting similar symptoms, such as amoebic dysentery, which is common among the targeted populations [10, 11]. The theoretical foundation in the Health Belief Model (HBM), integrates people’s knowledge, perceptions, attitude and practices to a disease in establishing trends of infection [12].

RETRACTED

The study further revealed a significant association (*p* ≤ 0.05) between washing of hands after visiting the toilet with having suffered from schistosomiasis infection. The current study was consistent with studies conducted in Gondar and Babile [12, 13], where there was significant association between intestinal parasitic infections and hand washing practice. A study conducted in Brazil reported that daily contact of open water source results in higher rate of infection by S. mansoni [14].

The current study indicates that, availability of toilet facility at home was significantly associated with having suffered from schistosomiasis infection. This does not concur with a study from Yemen which reported that the absence of a functioning toilet in the house was significantly associated with the prevalence of schistosomiasis and this was in accordance with other previous studies [15].

The findings of the present study showed that raring animals at home was significantly associated with having suffered from schistosomiasis infection. Results of a survey in Xinzhuang, indicated grazing cattle, digging vegetables, cutting grass in the field, and raising cattle by free grazing are some of the risk factors for schistosomiasis hence greater infection rates [16].

The study results further indicated that households being affected by floods was significantly associated with having suffered from schistosomiasis infection. While it is clear that sanitation breaks the transmission cycle of many diseases, the season can have impacts on the sanitation facilities themselves with heavy rains causing pit latrines and sewerage systems to flood and become inoperable and possibly contaminate the environment. A study by Wu XH et al. [17] indicated that the number of acute cases with schistosomiasis japonica was markedly higher in years characterized by floods; on average, 2.8 times more cases were observed when compared to years that the Yangtze River had normal water levels [17].

The present study reveal that gender, marital status, wearing protective gear and working in the rice paddies were not significantly associated with having suffered from schistosomiasis. This concurs with a study by Hany Sady et al. [18] which found no significant difference in the prevalence of schistosomiasis between male and female participants and marital status. The study indicated female as more prone to schistosomiaisis infection than men, these could be attributed to females being responsible for fetching water and washing clothes and utensils at these water sources, and therefore, have similar exposure to infective stages. Other studies elsewhere have also reported significantly higher infection rates among females compared to their males counterparts [19, 20].

RETRACTED

Self-protection during agricultural work plays an important role of reducing the risk of infection, at least in principal. However, this present study indicated no significance between wearing protective gear and having suffered from schistosomiaisis infection. This concurs with a study by which revealed that PPE wearing behaviours were not improved by the intervention that the project put in place. It still scored lowly. When asked about the reason for not using any protection, most people responded that “however useful in interrupting transmission, it was uncomfortable and inconvenient to wear rubber gloves or boots while working in the fields”. While this illustrates the difference between understanding the benefit and modifying behaviour, as suggested in other studies of occupationally-related behaviour change [21], it also raises the issue of the practicalities of sustained personal protection in an inherently risky environment. Spear et al. [22] argues that a focus on environmental improvements and monitoring systems to signal early risks of infection are better long-term solutions than personal protection in rural China as they are in occupational settings worldwide [22].

The study results reveal that working in the rice paddies was not significantly associated with having suffered from schistosomiasis. This does not concur with a study by Bukenya et al. [23] which indicated that schistosomiasis mansoni in the study area is closely linked to working in the rice paddies.

### Conclusions/significance

This study reveals inadequate knowledge, attitude and practices concerning schistosomiasis among the Mwea population, which could be a challenging obstacle to the endevour towards the elimination of schistosomiasis from Kenya. Schistosomiasis infection is still a major problem with regard to prevention and control in Mwea. Thus, there is a great need for a proper health education intervention and community mobilization in order to enhance prevention and instill better knowledge concerning the transmission and prevention of schistosomiasis. Providing efficient health education to people residing in schistosomiasis endemic areas is imperative for an effective and sustainable control programme in order to save the lives and future of the most vulnerable population in Kenya.

RETRACTED

These findings support an urgent need to start an integrated, targeted and effective schistosomiasis control programme with a mission to move towards the elimination phase. Besides periodic drug distribution, health education i.e. handwashing and community mobilisation, provision of clean and safe drinking water, introduction of proper sanitation are imperative among these communities in order to curtail the transmission and morbidity caused by schistosomiasis. Emergence response during floods should also be used as a mitigation strategy in curbing new infections. Screening and treating other infected family members should also be adopted by the public health authorities in combating this infection in these communities. This study recommends a focus on change in practices in the community to complement existing efforts aimed at creating knowledge and awareness on schistosomiasis.

### Study limitations

Since it was a Cross-Sectional study, it was therefore difficult to infer causality.

## Abbreviations

ESACIPAC: Eastern and southern Africa centre of international parasite control
FBOs: Faith based organizations
FGDs: Focus group discussions
HBM: Health belief model
JICA: Japan international cooperation agency
KAP: Knowledge attitude and practices
KEMRI: Kenya medical research institute
KIIs: Key informant interviews
SPSS: Statistical package for social sciences
STHs: Soil transmitted helminthes
WHA: World health assembly
WHO: World health organization
